The article "Modulation of immune cum inflammatory pathway by earthworm granulation tissue extract in wound healing of diabetic rabbit model" was retracted in 2025. Reasons: unreliable results or conclusions; concerns about the authorship.

# Modulation of immune cum inflammatory pathway by earthworm granulation tissue extract in wound healing of diabetic rabbit model

**DOI:** 10.1016/j.heliyon.2024.e24909

**Published:** 2024-01-27

**Authors:** Ahmed M. E. Elkhalifa, Sofi Imtiyaz Ali, Showkat Ul Nabi, Imran Bashir, Syed Taifa, Rabia Rakhshan, Iqra Hussain Shah, Muzafar Ahmad Mir, Masood Malik, Zahid Ramzan, Mehak Nazar, Nusrat Bashir, Shubeena Ahad, Ibraq Khursheed, Elham Elamin, Elsharif A. Bazie, Nasser A.N. Alzerwi, Musaed Rayzah, Bandar Idrees, Fares Rayzah, Yaser Baksh, Afnan Alsultan, Ahmed M. Alzahrani

**Affiliations:** a Department of Public Health, College of Health Sciences, Saudi Electronic University, Riyadh, 11673, Saudi Arabia; b Department of Haematology, Faculty of Medical Laboratory Sciences, University of El Imam El Mahdi, Kosti, 1158, Sudan; c Preclinical Research Laboratory, Department of Clinical Veterinary Medicine, Ethics & Jurisprudence, Sher-e-Kashmir University of Agricultural Sciences and Technology (SKUAST-Kashmir), Srinagar, J&K, 190006, India; d Department of Sheep Husbandry, Srinagar, Jammu & Kashmir, 190006, India; e Department of Clinical Biochemistry, University of Kashmir, Srinagar, Jammu & Kashmir, 190006, India; f Department of Zoology, Central University of Kashmir, 191201, Nunar, Ganderbal, Jammu & Kashmir, India; g Pediatric Department, Faculty of Medicine, University of El Imam El Mahdi, Kosti, 1158, Sudan; h Department of Surgery, College of Medicine, Majmaah University, P. O. Box 66, Al-Majmaah, 11952, Riyadh, Kingdom of Saudi Arabia; i Department of Surgery, Prince Sultan Military Medical City in Riyadh, Makkah Al Mukarramah Rd, As Sulimaniyah, Saudi Arabia; j Department of Surgery, Aseer Central Hospital, Abha, Saudi Arabia; k Department of Surgery, Al-Iman General Hospital, Riyadh, Saudi Arabia; l Department of Surgery, King Saud Medical City, Riyadh, Saudi Arabia

**Keywords:** Inflammatory markers, Wound healing, Wound healing markers and oxidative stress

## Abstract

Regeneration is a rare occurrence in the animal kingdom, but the earthworm stands out as a remarkable example of this phenomenon. Recent research has highlighted the promising wound healing properties of extracts derived from earthworms. Therefore, we propose that earthworm granulation tissue extract (EGTE) may facilitate wound healing by regulating immune responses in a rabbit diabetic wound model. Electron microscopy reveals that 70 % EGTE possesses noteworthy porosity with spherical to irregularly oval configuration. Gas chromatography–mass spectrometry (GC–MS) Characterization of EGTE revealed higher levels of ergosta-5,7,22-trien-3-ol, (3. beta.,22E). *In-Vitro* studies revealed significant anti-oxidant, anti-inflammatory and anti-bacterial properties in dose dependent manner. Likewise, cytotoxicity assessments reveal that 70 % EGTE exhibits minimal harm to cells while displaying substantial antioxidant and anti-inflammatory activities. For In-Vivo studies excision wounds were created on the dorsal regions of the experimental animals and were divided as Group I (50 % EGTE), Group II (70 % EGTE), Group III (vehicle) and Group IV (distilled water). Over a 21-day observation period 70 % EGTE facilitated the early healing of wounds in the experimental animals, evident through prompt wound closure, granulation tissue formation, increased DNA content, enhanced tensile strength of the wound area and enhanced the expression/synthesis of wound healing markers/proteins. From these results it can be postulated that EGTE accelerates wound healing by immune modulation, dampening of inflammatory pathway and enhanced expression of growth markers. Henceforth making it promising candidate for therapeutic use in diabetic wound healing.

The article "Modulation of immune cum inflammatory pathway by earthworm granulation tissue extract in wound healing of diabetic rabbit model" was retracted in 2025. Reasons: unreliable results or conclusions; concerns about the authorship.

## 1 Introduction

The skin, the body's largest organ, serves crucial functions such as thermoregulation, sensory perception, and acting as the primary defense against infections [1]. However, when this protective cutaneous barrier becomes compromised, it opens the door to a range of complications, including bacterial infections and loss of bodily fluids [2]. Beneath the skin's surface, a vast network of blood vessels exists, with most of them forming during fetal development. Nevertheless, adult tissues can stimulate the growth of new blood vessels, a process known as angiogenesis, in response to injury. This angiogenic response is governed by specific factors [3]. Within the spectrum of different wound types, diabetic wound healing is a dynamic process encompassing four interconnected phases: hemostasis, inflammation, proliferation, and epithelialization [4,5]. Diabetes, a metabolic disorder characterized by persistent hyperglycemia, is associated with various complications, including nephropathy, neuropathy, retinopathy, vascular dysfunction, and the development of diabetic ulcers [[6], [7], [8]]. Individuals diagnosed with diabetes face an increased risk of developing diabetic ulcers, a perplexing and highly distressing complication that further complicates their diabetes management [9,10]. The healthcare costs associated with treating these diabetic ulcers impose a substantial economic burden on patients, and these ulcers also exhibit a high recurrence rate, affecting approximately 50 % of diabetic individuals [11,12]. Researchers have identified several factors contributing to impaired diabetic wound healing, including reduced blood vessel formation, impaired skin cell regeneration, hindered fibroblast migration, and elevated levels of Tumor Necrosis Factor alpha (TNF-α) [13,14]. However, the exact mechanisms underlying delayed wound healing in diabetes remain incompletely understood. Recent studies have suggested that abnormal macrophage behavior and dysregulation of pro-inflammatory and inflammatory mediators play a central role in this delay [[15], [16], [17], [18]].

The article "Modulation of immune cum inflammatory pathway by earthworm granulation tissue extract in wound healing of diabetic rabbit model" was retracted in 2025. Reasons: unreliable results or conclusions; concerns about the authorship.

In previous decades, researchers have explored a wide range of herbal and traditional medicinal preparations derived from animals in lower phyla of the animal kingdom for their potential in diabetic wound healing [19,20]. These studies have reported promising results in wound healing for diabetic patients. Among these traditional remedies, various products and extracts derived from earthworms have demonstrated multiple pharmacological actions beneficial for promoting wound healing, including antioxidant properties and modulation of inflammatory pathways [21]. Additionally, these studies have noted that earthworm protein components can enhance the expression of genes involved in wound healing [22].

Numerous studies, encompassing both clinical and experimental investigations, have highlighted the role of oxidative stress and pro-inflammatory/inflammatory mediators in delayed wound healing in diabetes [23]. Although, there are few plant-based preparations (*Centella asiatica*) and mica based (Muscovitum) used for chronic wound healing, researchers have reported accelerated wound healing potential of these preparations [24,25]. But there are limited reports of these preparations being used for healing of diabetic wound. Furthermore, the bioactive profile of these preparations differs significantly from bioactive profile of EGTE [26], which provide wide spectrum of therapeutic choices/molecules for treatment of diabetic wound [27]. Given the rising prevalence of diabetes and the associated risk of diabetic ulcers, there is an urgent need to explore novel medications with minimal side effects. Recognizing the promising indications of wound healing potential in various earthworm-derived extracts and preparations [9,20], the current study was designed to assess the wound healing potential of earthworm granulation tissue extract in a rabbit model of diabetes induced by Streptozotocin (STZ). Furthermore, this study aimed to uncover and understand the mechanistic pathways facilitated by EGTE in wound healing in a diabetic rabbit model, with the ultimate goal of developing effective topical treatments for diabetic patients with wounds.

## 2 Material and methods

### 2.1 Preparation of earthworm granulation tissue extract

Earthworms (*Eisenia fetida*) were procured from authorized Vermi-compost center and these earthworms were acclimatized in laboratory animal section for seven days. On 8th day earthworms were washed with normal saline followed by washing with Phosphate-buffered saline (PBS). Head of the earthworm was recognized by its location in relation to clitellum (Fig. 1). Five hundred earthworms were amputated by surgical blade at 1/3rd length to tail as it has been reported that anterior part of clitellar segments regenerate following amputation [28]. After amputation earthworms were placed back in compost bags for three days for regeneration of amputated part (Fig. 1, Fig. 2). On 4th day post amputation earthworms were screened for regeneration (Fig. 1) and only those earthworms were selected in which regeneration tissue has developed. Following this about 1 cm of regenerated tissue was harvested from earthworms to prepare earthworm granulation tissue homogenate as per method of [21]. Briefly the regenerated tissue harvested was homogenized in Tris(hydroxymethyl)aminomethane hydrochloride (Tris-HCl) buffer (10 mM, pH 7.2) by mixing 1 part of regenerated tissue with four parts of buffer. The homogenate obtained was lyophilized as per method of [29]. Briefly, after homogenization of regenerated granulation tissue, the homogenate was stored in 2 ml plastic tubes which were placed at −80 °C to ensure sublimation. Sublimation process was monitored by placing temperature sensor in some of the randomly chosen tubes and after completion of sublimation process, dried tissues were smashed in tissue lyser by using stainless steel balls. The lyophilized earthworm granulation homogenate was preserved at −4 °C till its further use (Fig. 1, Fig. 2).

The article "Modulation of immune cum inflammatory pathway by earthworm granulation tissue extract in wound healing of diabetic rabbit model" was retracted in 2025. Reasons: unreliable results or conclusions; concerns about the authorship.

**Fig. 1:** (1A): Earthworms were collected with PBS (0.9 %), (1B): Identification of head region. (1C): Incision on anterior aspect. (1D): Identification of earthworms where granulation tissue has formed. (IE): Harvesting of granulation tissue from earthworms. (1F): Lyophilization of earthworm granulation tissue. (1G): Preparation of final preparation (EGTE).

**Fig. 2:** Schematic presentation of preparation of Earthworm Granulation Tissue Extract (EGTE), washed earthworms were cut on anterior end (1/3rd part). These earthworms were placed back in vermin-compost bags and after 3 days these earthworms were washed and granulation tissue developed were harvested and lyophilized.

### 2.2 Characterization of EGTE

#### 2.2.1 Morphology

Field Emission Scanning Electron Microscope (FESEM; TESCAN, USA) was utilized for evaluation of surface morphology of EGTE. These samples were sputter-coated with gold and images were taken at different magnifications. Liquid displacement method of (Purohit, ShivDutt et al., 2019) was used to calculate porosilty of EGTE as per following formula.

$$p\left(\%\right)=\frac{V1-V3}{V2-V3}\times 100$$

where p (%): indicates percentage porosity.

The article "Modulation of immune cum inflammatory pathway by earthworm granulation tissue extract in wound healing of diabetic rabbit model" was retracted in 2025. Reasons: unreliable results or conclusions; concerns about the authorship.

V1: Total volume of cylinder.

V2: Volume of cylinder after EGTE sample was placed in cylinder.

V3: Residual volume of cylinder after EGTE samples was removed.

#### 2.2.2 Elemental overlay of EGTE

Total elemental overlay was estimated by closed vessel microwave digestion followed by overlay analysis by Inductively Coupled Plasma Mass Spectrometry (ICP-MS). After fine grinding of EGTE, the aliquot was digested in concentrated nitric acid in closed vessel microwave system (CEM, Germany) at 160 °C. The filtrate so obtained was analyzed by ICP-MS in He-Mode.

#### 2.2.3 Identification of bioactive compounds

The sample preparation was performed by dissolving 20 mg EGTE in 2 mL High-performance liquid chromatography (HPLC) grade methanol and stirred continuously till the powder gets completely dissolved and solution was kept undisturbed for 3 h at room temperature, vortexed for 30.0 s followed by centrifugation at 3000 rpm for 5.0 min. The prepared sample was filtered through 0.45 μm PTFE filter before analysis. Final volume (1 mL) was used for Gas chromatography–mass spectrometry (GC- MS/MS) analysis. The identification of the compounds from the extract was performed on a capillary column (Agilent J & amp; W HP-5ms UI 30 m × 0.25 mm × 0.25 μm). Helium was used as carrier gas with the injector temperature 280 °C in split less mode. The oven program was operated at 70 °C (hold for 2.0 min) in the beginning, heated to 150 °C and then further heated to 200 °C and finally raised to 280 °C. The MS system was set in scan mode. The data interpretation was performed by Mass Hunter Qualitative Analysis Software (Sophia, Ande et al., 2022).

### 2.3 In-vitro anti-inflammatory and anti-oxidant and anti-microbial assay

#### 2.3.1 in-vitro anti-oxidant assay

In-vitro anti-oxidant assay of EGTE was conducted by 2,2-diphenylpicrylhydrazyl (DPPH) assay and H_2_O_2_ assay as per the standard procedure of (Syed Muntazir Andrabi et al., 2020). Briefly three concentrations (50 %, 70 % and 100 %) of EGTE were incubated in DPPH (100 μM) and hydrogen peroxide (100 μM) for 90 min under dark environmental conditions. Following the incubation, the absorbance of these samples was measured at 517 nm. For measuring absorbance of standard and blank equal volume of methanol was used as standard and equal volumes of H_2_O_2_/DPPH were used as blank. Antioxidant activity of EGTE was measured as following

$$\text{Antioxidant}\;\text{Activity}\;(\%=\frac{Absorbance\;of\;control-Absorbance\;of\;sample\;}{Absorbance\;of\;control}\times 100$$

The article "Modulation of immune cum inflammatory pathway by earthworm granulation tissue extract in wound healing of diabetic rabbit model" was retracted in 2025. Reasons: unreliable results or conclusions; concerns about the authorship.

#### 2.3.2 In-vitro anti-microbial assay

For anti-microbial assay, disc diffusion method was followed. Briefly, loopful of test micro-organisms were inoculated on nutrient agar petri dishes and incubated until colonies become apparent. Following this, test substances, positive and negative control were placed over nutrient agar petri dishes and incubated for 24 h. After 24 h diameter of the clear zone (zone of inhibition) around the test substances were measured as per standard procedure [30].

#### 2.3.3 In vitro anti-inflammatory activity

Rabbit Red Blood Cells membrane integrity estimation was used to evaluate in-vitro anti-inflammatory activity (Gandhisan et al., 1991). 5 ml of collected blood was mixed with equal volumes of 50 % EGTE, 70 % EGTE, 100 % EGTE, 0.98 % Nacl (Sodium chloride) (negative control) and deionized water (positive contro). These assay mixtures were incubated at 37 °C for 4 h and after that these samples were centrifuged for 10 min @ 1500 rpms and supernatants were collected and absorbance were measured at 545 nm (Singh, Hemant et al., 2020).

$$\text{Hemolysis}\;\left(\%\right)=\frac{OD\;\left(EGTE\right)-OD\;\left(Negative\;Control\right)\;}{OD\;\left(Positive\;Control\right)-OD\;\left(Negative\;Control\right)}\times 100$$

#### 2.3.4 Cytotoxicity assay

Earthworm granulation tissue extract was evaluated for cytotoxicity assay using L929 cells. EGTE at three different concentrations (50 %; 70 % and 100 %) were placed in tissue culture plates and these plates were subsequently seeded with L929 cells @ 5000 cells/cm^2^. The whole procedure was conducted under sterile conditions. These plates (with or without EGTE) were cultured in Dulbecco's Modified Eagle Medium (DMEM) and were incubated at 37 °C under humidified 5 % CO_2_ for 24 h. After 2nd, 5th and 8th hour of incubation cells were trypinised and cell count was estimated by hemocytometer. Furthermore, proliferation assay was conducted on 1st, 3rd and 5th day after incubation using 3-[4,5-dimethylthiazol-2-yl]-2,5 diphenyl tetrazolium bromide (MTT) assay. For MTT assay Medias were removed on predetermined interval and were washed with PBS and subsequently 50 μl of MTT dye @ 5 mg/ml in PBS were added to each tube and these tubes were incubated for 4 h. Following this solubilization buffer Dimethyl sulfoxide (DMSO) was added to tubes and these plates were observed for absorbance at 540 nm. For assessment of cell viability, L929 cells were stained with fluorescein diacetate/ethylene dibromide for 5 min at 37 °C and were observed under florescent microscope to calculate dead/live cell percentage (Singh, Hemant et al., 2020).

The article "Modulation of immune cum inflammatory pathway by earthworm granulation tissue extract in wound healing of diabetic rabbit model" was retracted in 2025. Reasons: unreliable results or conclusions; concerns about the authorship.

### 2.4 Laboratory animals

Present study design was approved by institutional ethical committee faculty of veterinary sciences and animal husbandry, SKUAST-K (FVSc/VCC-9/19/439-40). Total of 30 Himalayan rabbits (3 months old) weighing between 2.5 kg and 2.7 kg were purchased from authorized Government Rabbit Breeding Farm. Seven days prior to experiment rabbits were allowed to acclimatize in laboratory animal house under standard environmental conditions (22–25 °C and a 12-h light/dark cycle). On 8th day animals were kept for overnight fasting and on morning of 9th day diabetes was induced by single intra-peritoneal injection of streptozotocin (STZ) @ 60 mg/kg body weight in phosphate buffer (pH-7.2). For next four days, these rabbits were screened for diabetes induction and only those rabbits were further included in experimental design in which diabetes has been successfully induced (Fig. 3, Fig. 4). In present study blood glucose level above 250 mg/dl were considered hyperglycemic suggestive of diabetes mellitus.

**Fig. 3:** (3A, 3B, 3C) Preparation of dorsal region of rabbit model for induction of wound, (3D, and 3E) surgical induction of wound. Application of different topical preparations on rabbits of different groups with follow up for 21 days. (3G) Representative remaining unhealed area on 0^th^ day (orange) 3rd day (Black) and 21st day (Red).

**Fig. 4:** Schematic representation of experimental design, after 7 days of acclimatization, diabetes was induced, on 12th day animals were screened for diabetes mellitus and animals found positive went for surgical induction of full thickness wound on 13th day. Following this animal were divided into four groups and were evaluated for healing process.

### 2.5 Dermal allergic response

For allergic dermal response three rabbits were randomly selected and dorsal region of these rabbits were shaved and 2 ml of EGTE with highest concentration (70 %) were applied topically. The site on which EGTE was applied was observed at periodic intervals of 24th, 72nd and 94th hour. In above three subjects no sign of irritation/adverse reaction was observed. All three animals were active and their behavior was normal with no mortality observed during study period of 92 h.

### 2.6 Experimental design

On 5th day post STZ injection, animals were screened for successful induction of diabetes mellitus and only those animals were included in present study in which diabetes was successfully induced (n = 24). All diabetic rabbits were wounded on 6th day post STZ injection, full thickness wounds with size of 2 cm^2^ were made on back in each rabbit as per method of [31]. Briefly the rabbits were anesthetized with intravenous injection of ketamine (100 mg/kg body weight). Dorsal region of rabbits was prepared by shaving hairs followed by application of disinfectant (70 % ethanol). On the dorsolateral right and left side (1:1) of the back, 2 mm × 2 mm area was marked with sterile ink and dermal tissue within the marked area was removed precisely by means of surgical blade (No. 18) to create full thickness skin wound having depth of 1.2 ± 0.4 cm. the full thickness skin wound was created precisely sparing the underlying muscular layer (Fig. 3) and regular disinfection procedures was followed throughout the experiment by applying 2 % povidone iodine on wound surface once a day.

The article "Modulation of immune cum inflammatory pathway by earthworm granulation tissue extract in wound healing of diabetic rabbit model" was retracted in 2025. Reasons: unreliable results or conclusions; concerns about the authorship.

After induction of wound, treatment was followed as per Table 1. These rabbits were divided into four groups (n = 6; 3 with right dorsolateral and 3 with left dorsolateral wound) and were treated with different topical formulations to evaluate wound healing potential of earthworm granulation tissue preparation. Briefly wound I was treated with 50 % lyophilized earthworm granulation tissue preparation; wound II was treated with 70 % lyophilized earthworm granulation tissue preparation, wound III was treated with ointment base (phosphate buffer saline) and wound IV was treated with distilled water. Each wound was treated with these formulations for seven days once daily (Fig. 3, Fig. 4). On 3rd, 7th and 14th day post induction of wound observational study of wound and collection of granulation tissue developed from wounded area was conducted as per method of [28]. Briefly each wound was photographed and wound area/percentage of wound contraction was calculated.

**Table 1:** Experimental design for evaluation of wound healing potential of EGTE at different doses in rabbit model.

Group	Treatment
Wound I	Treated with 50 % earthworm granulation tissue preparation.
Wound II	Treated with 70 % earthworm granulation tissue preparation
Wound III	Treated with ointment base (phosphate buffer saline)
Wound IV	Treated with distilled water

#### 2.6.1 Identification of biochemical/molecular markers of wound healing in rabbit model

For identification of molecular factors that promote/retard wound healing, in present study we attempted to compare biochemical/molecular markers with rate of wound healing in rabbit model by correlation matrix analysis. The parameters which exhibited positive/negative correlation with rate of wound healing were identified; henceforth the role of EGTE was evaluated in rabbit model based on dynamic changes in these identified promoters and inhibitors of wound healing.

#### 2.6.2 Estimation of anti-oxidative stress markers and pro-inflammatory markers in granulation tissue

Anti-Oxidant stress parameters were analyzed in wet granulation tissue samples as per method of [32]. The anti-oxidant markers analyzed included superoxide dismutase (SOD), Catalase, lipid peroxidation (LPO), reduced glutathione peroxidase (GSH), Nitric oxide (NO), Vitamin C and glutathione peroxidase (GPx). The pro-inflammatory markers which include Interleukins (IL), IL-1, IL-2, IL-6 and TNF- α were estimated in granulation tissue of animal model as per method of [33,34].

The article "Modulation of immune cum inflammatory pathway by earthworm granulation tissue extract in wound healing of diabetic rabbit model" was retracted in 2025. Reasons: unreliable results or conclusions; concerns about the authorship.

#### 2.6.3 Estimation of connective tissue parameters

Granulation tissue samples collected on different time intervals was dried at 50 C for 24 h. These dried samples were used for estimation of connective tissue parameters as per the method of [16]. The connective tissue parameters estimated in present study included Hydroxyproline (HPR), Hexosamine (HXA) and Hexuronic acid (HUA).

#### 2.6.4 Growth markers

The Deoxyribonucleic acid (DNA) content in granulation tissue were estimated as per method of [31]. Gene expression of growth factors was determined as per method of [35]. Tissue samples collected at 5th day of healing were analyzed for concentration of growth factors. In current study we analyzed granulation tissue for messenger ribonucleic acid (*m*-RNA) expression of Epidermal Growth Factor (EGF), Transformational Growth Factor 1-Beta (TGF-1β) and Vascular Endothelial Growth Factor (VEGF). Briefly, RNA was extracted from granulation tissue and reverse transcribed to produce complementary DNA (c-DNA) library and primers were purchased from authorized laboratory. The expression of these marker genes was normalized to housekeeping gene glyceraldehyde-3-phosphate dehydrogenase (GAPDH) using the 2- ^ΔΔCt^ method. The primer sequences of growth factors considered in present study are indicated in Table 2.

**Table 2:** Primer sequences of EGF, TGF-1β and VEGF used for expression studies of growth markers to evaluate wound healing potential of EGTE at different doses in rabbit model.

S. No	Genes	Forward primer	Reverse primer
1.	Epidermal Growth Factor (EGF)	5′-GCACAACACAGATGGAAGCAG-3′	5′-CCCTTTTTGGTGACCGTATCT3′
2.	Transformational Growth Factor 1-Beta (TGF-1β)	5′-AAGGGCTACCACGCCAACTT-3′	5′-CCGGGTTGTGCTGGTTGTAC-3′
3.	Vascular Endothelial Growth Factor (VEGF)	5′-GTGGACATCTTCCAGGAGTA-3′	5′-GGTCTGCATTCACATTTGTTG-3′

#### 2.6.5 Histopathology

Punch biopsy was conducted at different time intervals of 0^th^ day, 3rd day and 7th day post induction of wound. The samples were fixed with 10 % formalin for 21 days. Samples submitted to histopathology section were stained with hematoxylin-and-eosin (H&E) and samples were processed as per method of [36,37].

The article "Modulation of immune cum inflammatory pathway by earthworm granulation tissue extract in wound healing of diabetic rabbit model" was retracted in 2025. Reasons: unreliable results or conclusions; concerns about the authorship.

### 2.7 Statistical analysis

The present study was designed to evaluate efficacy of earthworm granulation tissue extract in management of diabetic wound. Primary outcome of current study was to estimate the reduction of wound area using mixed effect model. Qualitative variables were analyzed by chi square test and data was presented as odds ratio with 90 % confidence interval (CI). Quantitative variables were analyzed using Shapiro–Wilk test as data in present study was normally distributed. To evaluate differences between different treatment groups Kruskal-Wallis test was used. For above statistical test level of statistical significance was set at P < 0.05. Statistical analysis was performed as per method of [38].

## 3 Results

### 3.1 Characterization of EGTE

#### 3.1.1 Morphology

SEM images of 50 % EGTE and 70 % EGTE showed presence of almost spherical and non-aggregated droplets. Images of EGTE when investigated using Image J analysis, revealed particle size of EGTE ranging from 667 μm to 1879 μm with porosity of 45 % (Fig. 5a, b and 5c).

**Fig. 5:** Characterization and physiochemical properties of EGTE: (a) FESEM image of 50 % EGTE (b) FESEM image of 70 % EGTE (c) porosity of different formulation (d,e) elemental overlay/profile (f) GC-MS profile(*p˂0.05).

#### 3.1.2 Elemental overlay

Many elements have been recognized to play an important role in wound healing and hence current research supports elemental profiling of the various plant and animal-based extracts. Elemental profiling of EGTE revealed presence of magnesium, iron copper and zinc which are supposed to play significant role in wound healing process owing to their antimicrobial, anti-inflammatory and anti-oxidant activities. Hence from elemental profiling it may be postulated that these elements present in EGTE have significant role to play in wound healing (Fig. 5d and e).

#### 3.1.3 Bioactive components of EGTE

GC-MS has been found to be an efficient method for evaluation of bioactive components present in biological samples and other bioactive extracts obtained from biological sources. GC-MS chromatograph of EGTE showed peaks which corresponds to presence of 58 bioactive components. The bioactive components with their retention time, molecular weight and other associated characteristics are shown in Supplementary Table 1. Among the 58 compounds identified in EGTE, 7 were heptane derivatives and 12 were octadecadienoate derivatives with more than 15 carbon atoms, while rest of the components identified included molecules with less than 10 carbon atoms, with at least one methyl group attached with molecular core. The bioactive components with ascending order of retention time are indicated in Supplementary Table 1 and Fig. 5f. The compounds present in highest amount were ergosta-5,7,22-trien-3-ol, (3.beta.,22E) (RT-12.019; 35.81 %) followed by diethyl phthalate ergosta-5,8–dien-3-ol, (3.beta) (RT-34.58; 8.12 %), 6,7-Dimethoxy-1,4-dimethyl-1,4-dihydro-2,3-quinoxalinedithione (RT-39.80; 4.16 %), and Tris (*tert*-butyl dimethyl silyloxy) arsane(RT-34.87; 2.99 %) (Fig. 5f; Supplementary Table 1).

The article "Modulation of immune cum inflammatory pathway by earthworm granulation tissue extract in wound healing of diabetic rabbit model" was retracted in 2025. Reasons: unreliable results or conclusions; concerns about the authorship.

### 3.2 In vitro analysis

#### 3.2.1 In vitro cytotoxicity assessment

Fig. 6a and b shows hemocompatibility of EGTE at different concentrations with their capability to cause protection against hemolysis. In present study we found 50 % and 70 % concentration of EGTE compatible with red blood cells, while as 100 concentration was found to cause significant hemolysis compared to other two concentrations. Furthermore, L929 fibroblasts were found to proliferate in presence of all concentrations of EGTE, which is reflected by increased OD values on 1st, 3rd and 5th day. An interesting finding obtained from present study indicated increased OD values of 70 % concentration of EGTE was found to vary significantly compared to OD values of other two concentrations. Similarly values of OD for respective concentrations were found to increases significantly on 3rd and 5th day compared to OD values on 1st day. On 3rd day, Live/dead cells observed across different time intervals were found to have significantly higher live cells (93.18 %) in 70 % EGTE concentration compared to live cells observed in other two concentrations. Similarly, on 5th day live cells were found to overpopulate compared to dead cells in all formulated concentrations (Fig. 6c).

**Fig. 6:** *In-Vitro* characterization of EGTE: (a) cytotoxicity assay of EGTE (b) MMT assay of EGTE (c) cellular proliferation assay (d) H_2_O_2_ assay of EGTE exhibiting antioxidant activity against H_2_O_2._ (e) DPHH assay showing antioxidant activity of EGTE(*p˂0.05; **p˂0.01; *** (*p˂0.001). (f and g) In-Vitro anti-microbial assay depicting significantly higher zone of inhibition around 70 % EGTE compared to 50 % EGTE while as zone of inhibition around penicillin was significantly higher compared to 50 % and 70 % EGTE.

#### 3.2.2 In-vitro antioxidant and anti-microbial properties

Fig. 6d and e indicates DPPH based oxidants that are scavenged by EGTE formulations. The formulations exhibited dose dependent decline in free radical levels with sharp decline observed in 100 % EGTE. These three formulations exhibited significant differences compared to negative control. Similarly, H_2_O_2_ assay revealed free radical scavenging activity of EGTE formulations in dose dependent manner. In-vitro antioxidant activities observed in H_2_O_2_ assay were almost similar to DPPH assay (Fig. 6d and e). EGTE showed potent anti-bacterial activity against reference gram-positive (S. aureus) and gram-negative (E. coli) bacteria in dose dependent manner. 70 % EGTE showed significantly higher anti-bacterial activity compared to 50 % EGTE Furthermore both 50 % EGTE and 70 % EGTE showed most potent and significant anti-bacterial activity compared to Distilled water and Vehicle Control (Fig. 4a and b).

The article "Modulation of immune cum inflammatory pathway by earthworm granulation tissue extract in wound healing of diabetic rabbit model" was retracted in 2025. Reasons: unreliable results or conclusions; concerns about the authorship.

#### 3.2.3 In-vitro anti-inflammatory activity

EGTE was investigated for in-vitro anti-inflammatory action by measuring hemolysis assay and protection offered by extracts against hemolysis. The 70 % EGTE showed maximum protection and minimum hemolysis in hypotonic solution. Results of present study indicate erythrocyte membrane stabilization activity of EGTE, which indicates its possible stabilization of lysosome membrane which limits release of lysosome constituents which are important mediators of inflammation. Hence from these results it can be postulated that EGTE possess anti-inflammatory action at 70 % concentration, henceforth shortens the inflammatory phase of wound healing which promote wound healing (Fig. 6a).

### 3.3 Relationship between wound healing and biochemical/molecular response in rabbit model

In order to identify role of biochemical/molecular response in rabbit model, present study attempted to evaluate correlation between biochemical/molecular response and rate of healing (% of healing) in rabbit model. From these correlation studies we found significant correlation between rate of healing and levels of VGEF (y = 1.56 x + 198.2; r^2^ = 0.81; p < 0.05), TGFβ1 (y = 0.831x + 208.1; r^2^ = 0.70; p < 0.05), EDGF (y = 1.19x + 172.5; r^2^ = 0.74; p < 0.05), Hexosamine (y = 1.34x + 119.8; r^2^ = 0.65; p < 0.05), Hydroxyproline (y = 0.780x + 334.8; r^2^ = 0.64; p < 0.05) and Hexuronic acid (y = 1.23x + 102.5; r^2^ = 0.59; p < 0.05), IL-2. On similar line, ILs (IL‐2, and IL‐4), NO inhibition and Catalase levels showed significant positive correlation with healing rate in rabbit model (Fig. 7). Contrarily, present study found negative correlation in TNF-α (y = 2.56x + 178.7; r^2^ = −0.43; p < 0.05), LPO (y = 1.59x + 264.6; r^2^ = −0.80; p < 0.05) and IL-6 (y = 1.59x + 151.5; r^2^ = −0.46; p < 0.05) with healing rates in rabbit model. Henceforth in subsequent parts of present study, we compared these parameters in animals undergoing different topical treatment. In current experimental design we evaluated wound healing potential of earthworm granulation tissue extract in rabbit model. The wound healing potential in present study was evaluated on basis of anti-oxidants, pro-inflammatory cytokines, connective tissue markers and growth markers which are considered as hallmarks for evaluation of wound healing properties of test extracts and we attempted to highlight those markers in present study which showed significant role in wound healing process as can be appreciated from correlation studies (Fig. 7) [1,2,6,7,23].

The article "Modulation of immune cum inflammatory pathway by earthworm granulation tissue extract in wound healing of diabetic rabbit model" was retracted in 2025. Reasons: unreliable results or conclusions; concerns about the authorship.

**Fig. 7:** Heat plot matrix to find correlation (Pearson's correlation) between percentage of wound healing and other parameters considered in present study.

### 3.4 Gross findings

In present study on full thickness skin wound, percentage of wound contraction in group III was 58 % on 14th day and complete closure of wound (epithelization) was observed on 27th day. In group IV 67 % of wound closure on 14th day and complete wound healing was observed on 22nd day. In group I 79 % epithelization was observed on 14th day and complete wound healing was observed on 20th day. Similarly, the accelerated rate of wound healing was observed in wound II as 82 % closure of wound was observed on 14th days and complete closure of wound was observed on 18th day. Furthermore, granulation tissue development was evident from significant increase in wet weight of granulation tissue per 100 g body weight as significantly higher levels (P < 0.01) of granulation tissue (mg)/100 gms body weight was observed in group I (102.56 ± 12.16) and group II (145.45 ± 23.56) compared to group III (73.67 ± 12.34) and group IV (54.67 ± 23.34). The gross findings/appearance of wounds observed in animals of different groups is described in Table 3 and Fig. 3. In order to evaluate whether EGTE promotes wound healing in diabetic laboratory animals, wound area was calculated on 0^th^, 3rd, and 7th day after application of different topical therapeutic interventions. Up to 3rd day no significant difference was observed in contraction of wound edges across different treatment group (21 % in 50 % EGTE group; 19 % in 70 % EGTE group; 24 % in Vehicle control Group and 22 % in Distilled Water Group). while as on 7th day significant difference was observed between wound closure area in 70 % EGTE group (91 %) and 50 % EGTE group (87 %) compared to vehicle control group (35 %) and Distilled water Group (42 %) (Fig. 3). Further, from Table 3 and Fig. 3 it can be seen that EGTE modulated inflammatory response effectively and wound edges in EGTE groups were found to be well defined and clear which support their role in healing process of diabetic wound. On 3rd day we isolated granulation tissue for biochemical analysis, the granulation tissue isolated was subjected to evaluation of pro-inflammatory cytokine response, connective tissue markers, anti-oxidant markers, and growth factor markers which are described below.

The article "Modulation of immune cum inflammatory pathway by earthworm granulation tissue extract in wound healing of diabetic rabbit model" was retracted in 2025. Reasons: unreliable results or conclusions; concerns about the authorship.

**Table 3:** Gross findings of wound examined after application of different therapeutic protocols, the findings observed included degree of inflammation, appearance of wound edges, granulation tissue and presence and type of exudates.

Groups	Degree of inflammation	Appearance of Wound edges	Appearance of granulation tissue	Presence and type of exudates
**EGTE (50 %)**	Redness present with no discharge	well defined not attached to wound base and thickened	bright beefy red, 75 %–25 % wound filled	scant, wound base moist and no measurable exudates
**EGTE (70 %)**	Clean wound	well defined fibrotic and scarred	bright beefy red, 75–100 % wound filled	small, wound tissue moist and moisture evenly distributed
**Vehicle control**	redness, swelling and discharge present	indistinct, diffuse and outline not visible	No granulation tissue	Large, wound tissue bathed in fluid.
**Distilled water**	Redness present with no discharge	well developed not attached to wound based	pink or dull red, less or equal to 25 % of wound healed	moderate, wound base saturated

### 3.5 Oxidative stress parameters

There are plethora of studies that have reported beneficial role of anti-oxidants in wound healing process; therefore it can be proposed that drugs/herbal remedies that ameliorate oxidative stress will be having therapeutic role in wound healing process. Keeping in view these facts, evaluation of anti-oxidant molecules in granulation tissue formed were estimated which revealed significantly higher levels of antioxidant potential in granulation tissue treated with EGTE (group I and II) compared to control groups (group III and IV) (Fig. 8). GSH levels were found to be significantly (P < 0.0001) elevated in group I (27.67 ± 1.56 mmol/mg) and group II (32.67 ± 2.45 mmol/mg) compared to group III (17.56 ± 1.23 mmol/mg) and group IV (14.98 ± 1.89 mmol/mg). On similar lines SOD levels were found to be increased in EGTE groups (group I-23.45 ± 4.72 U/mg; group-II 16.78 ± 5.12 U/mg) compared to levels in control groups (group III-11.45 ± 4.23 U/mg; group IV-9.44 ± 2.87 U/mg), Levels of SOD were almost twice in group II compared to levels in control groups. Comparing levels of catalase, EGTE treated groups were found have nearly threefold (67.78 ± 12.34 mmol/mg in group II and 45.89 ± 7.45 mmol/mg in group I) increased level compared to levels in control groups (22.33 ± 7.87 mmol/mg in group III and 15.89 ± 3.77 mmol/mg in group IV). Furthermore, EGTE treated groups (45.67 ± 12.34 % in group-I and 56.78 ± 15.87 % in group II) showed significant increase in nitric oxide (NO) inhibition compared to control groups. Contrarily to these findings free radical mediated cellular damage marker (LPO) levels were significantly decreased in EGTE treated groups compared to control groups. From these findings specifically decreased levels of LPO and NO contents indicate an effective role of EGTE in prevention and amelioration of damage mediated by free radicals which henceforth dampens the activation of inflammatory pathways which promotes accelerated healing process.

The article "Modulation of immune cum inflammatory pathway by earthworm granulation tissue extract in wound healing of diabetic rabbit model" was retracted in 2025. Reasons: unreliable results or conclusions; concerns about the authorship.

**Fig. 8:** Comparison of oxidative stress parameters of granulation tissue harvested from rabbits after application of different ointments in different experiment groups, comparison was made at levels of (p˂0.05: p˂0.001).

### 3.6 Pro-inflammatory cytokines

On 5th day of induction of wound, ILs and TNF‐α responses of laboratory animals were compared with ILs and TNF‐α responses on 2nd day in four treatment arms. In present study we could not find any significant difference between IL-4 levels on 2nd and 5th day across four treatment groups (Fig. 9). On 5th day significant reduction was observed in levels of IL-6 in a dose dependent manner, on 5th day IL-6 levels in EGTE (50 %) group and vehicle control group were significant (p < 0.05) reduced compared to levels on 2nd day post induction of wound, similarly in EGTE (70 %) group more pronounced reduction in levels of IL-6 were observed (p < 0.01), while non-significant reduction was observed in distilled water group. When we compared levels of TNF-α across different treatment groups on 2nd and 5th day post induction of wound, significant reduction in levels of TNF-α were observed in EGTE (50 %) group (p < 0.05) and EGTE (70 %) group (p < 0.05). Furthermore, in present study we could not observe any significant difference in levels of TNF-α across 2nd and 5th day in vehicle control group and distilled water group. Furthermore on 5th day dose dependent significantly elevated levels of IL-1 were observed in EGTE (50 %) group (p < 0.05) and EGTE (70 %) group (p < 0.01). Vehicle control group showed non-significant increase in IL-1 levels on 5th day compared to levels on 2nd day of wounding, in addition to this in distilled water group levels of IL-1 remained more or less same. On similar lines when present study compared levels of IL-1α across different treatment arms on 3rd and 5th day, only EGTE (70 %) group showed significant (p < 0.05) reduction in levels of IL-1 α on 5th day compared to levels on 2nd day of wound induction.

**Fig. 9:** Comparison of pro-inflammatory markers in blood on 2nd and 5th day after application of different ointments in different experiment groups, comparison was made at levels of (p˂0.05: p˂0.001).

The article "Modulation of immune cum inflammatory pathway by earthworm granulation tissue extract in wound healing of diabetic rabbit model" was retracted in 2025. Reasons: unreliable results or conclusions; concerns about the authorship.

### 3.7 Connective tissue markers

In current study connective tissue markers in granulation tissue formed on 3rd day in experimental rabbits were compared between control groups and interventional groups. Connective tissue parameters compared in present study revealed that wounds treated with EGTEs (50 % and 70 %) showed significantly increased levels of connective tissue markers compared to control group and distilled water group (Fig. 10). The wound healing properties of EGTE were found to be effective in dose dependent manner in EGTE groups. In dried granulation tissue significantly higher levels of hydroxyproline were observed in group I (EGTE-50 %) (47.80 ± 13.21 mg/g) and group II (EGTE-70 %) (56.90 ± 21.80 mg/g) compared to levels found in group III (Vehicle control) (23.89 ± 6.56 mg/g) and group IV (Distilled Water) (21.67 ± 7.89 mg/g). Similar trend of increased levels of Hexosamine and Hexuronic acid was observed in different interventional groups of present study, where levels of Hexosamine and Hexuronic acid were almost three-fold increased in EGTE groups compared to levels in group III and group IV. Interestingly, levels of all connective tissue markers were in dry granulation tissue were observed to be elevated this indicates wound healing properties of EGTE via synthesis and stabilization of collagen fiber.

**Fig. 10:** Comparison of connective tissue markers in granulation tissue of rabbits harvested after application of different ointments in different experiment groups, comparison was made at levels of (p˂0.05: p˂0.001).

### 3.8 DNA concentration in granulation tissue and growth markers

DNA content in granulation tissue gives an indirect indication about wound healing potential of different tropical preparations. In present study when DNA content was compared in different diabetic animal groups, EGTE (70 %) and EGTE (50 %) showed significantly elevated DNA content compared to control and vehicle group. Among entire experimental groups of present study EGTE (70 %) group showed maximum content of DNA which reflects role of EGTE in promotion of DNA synthesis and henceforth its role in synthesis of macro-molecules for new cellular and extracellular framework (Fig. 11). When the experimental rabbits in EGTE groups (70 % and 50 %) were compared with distilled water and vehicle group for gene expression of growth promoters which include TGF-β1, IGF-I, and EGF. EGTE groups (70 % and 50 %) were found to cause increased expression of TGF-β1, IGF-I and EGF mRNA (p < 0.05) compared to expression of these genes in vehicle and distilled water group. In addition to these findings, from Fig. 11 it can be seen that EGTE caused enhanced expression of TGF-β1, IGF-I and EGF in dose dependent manner. From these findings it can be postulated that this difference could be because EGTE promotes expression of these markers and hence promotes wound healing process.

The article "Modulation of immune cum inflammatory pathway by earthworm granulation tissue extract in wound healing of diabetic rabbit model" was retracted in 2025. Reasons: unreliable results or conclusions; concerns about the authorship.

**Fig. 11:** Evaluation of expression of growth markers (RNA) in granulation tissue harvested from rabbits in different experiment groups, comparison was made at levels of (p˂0.05: p˂0.001).

### 3.9 Histopathology

Histopathological studies of granulation tissues isolated on 3rd and 5th day post induction of wound were conducted to evaluate role of EGTE in wound healing process. On 3rd day in vehicle control group and distilled water group, present study observed widespread infiltration of mononuclear inflammatory cells and fibroblasts in proliferating granulation tissue which indicates prolongation of inflammatory phase of healing in these groups. On 5th day, although degree of mononuclear inflammatory cells infiltration was reduced compared to levels on 3rd day but still levels of cellular infiltration were more than levels observed in EGTE groups. The rabbits treated with EGTE displayed pronounced abundance of collagen deposition and little inflammatory cell infiltration compared to controls groups on 3rd and 5th day, which indicates profound role of EGTE in wound healing. As can be seen from Fig. 12 distinctive histopathological changes of wound samples were found on 3rd and 5th day post induction of wound between EGTE groups and control groups (vehicle and distilled water). Thin layer of primary epidermis was well formed in EGTE groups on 3rd day, which indicates proliferative stage of wound healing. However, in control groups only thick layer of scar with numerous inflammatory cells were found which indicates inflammatory phase of wound healing.

**Fig. 12:** Histopathological examination of granulation tissue harvested from rabbits in different experiment groups, these figures indicate well defined neo-epidermis in group EGTE (50 % and 70 %) while scar was persistent in vehicle and distilled water group.

## 4 Discussion

In present study, we successfully demonstrated wound healing properties of EGTE in rabbit model via gross findings, oxidative stress, connective tissue markers, pro-inflammatory markers and expression of growth markers which are considered as most important parameters for medicinal preparations having wound healing potential [7,9,11]. In recent times researchers have proposed that biomedical preparations obtained from biologics having abundant concentration of growth factors can accelerate wound healing in diabetic patients [13]. Chromatographic characterization revealed presence of ergosta class of active principles [ergosta-5,7,22-trien-3-ol and diethyl phthalate ergosta-5,8–dien-3-ol, (3. beta)] present in highest proportion in EGTE. There are number of earlier studies that have reported immunomodulatory effect of compounds belonging to ergosta family of compounds [[39], [40], [41]]. These compounds activate nuclear factor erythroid 2-related factor 2 (Nrf2) signaling, henceforth modulating immune response [41]. Likewise, studies have reported that ergosta family of compounds cause attenuation of mitogen-activated protein kinase/activator protein-1 (MAPK/AP-1) pathway and interleukin-6/Janus kinase/signal transducer and activator of transcription (IL-6/JAK/STAT) pathway which results in modulation of immune cum inflammatory pathways [39,42,43]. In addition to this JAKs are cytoplasmic tyrosine kinases that could phosphorylate and dimerize the STATs, these dimerized entities are translocated to nucleus and bind with DNA which causes selective expression of genes responsible for immune activation. Contrarily to this addition of ergosta class of active principles results in transcriptional blockage of these genes and hence results in immune modulation [44,45].

The article "Modulation of immune cum inflammatory pathway by earthworm granulation tissue extract in wound healing of diabetic rabbit model" was retracted in 2025. Reasons: unreliable results or conclusions; concerns about the authorship.

To best of our knowledge, there are very limited numbers of studies that have evaluated wound healing potential of EGTE extracted from anterior end of regenerating earthworm tissue. Although there are some earlier studies that have reported wound healing potential of earthworm coelomic fluid and tissue extracts of earthworm [20], but these studies have not gone into depth to understand the role of different molecular/biochemical markers in wound healing. Our results demonstrate that topical application of EGTE accelerates acute wound healing in diabetic rabbit model and anti-oxidant enzymes, connective tissue markers and growth promoter genes play prominent role in this process. Taken together these all changes results in regulation of immune pathways and shorten the inflammatory phase of wound healing which promotes wound healing [5,46,47]. Although, there are some studies that have reported therapeutic superiority of diabetic wound healing by hydrogel-based preparations [5,46,47]. The advantage that current study offer over these studies includes that some preparations being injectable [46], which need expertise for administration. Furthermore, these preparations have different biochemical profile compared to EGTE and further research can be designed keeping earlier studies [46,47] in consideration with current study to fabricate therapeutically efficient wound healing preparations for diabetic patients. Likewise, these studies [5,46,47] and current study depicts wide spectrum of biologically active molecules that can be evaluated for synergistic activity for diabetic wound healing.

The article "Modulation of immune cum inflammatory pathway by earthworm granulation tissue extract in wound healing of diabetic rabbit model" was retracted in 2025. Reasons: unreliable results or conclusions; concerns about the authorship.

After successful formulation of EGTE, the morphological characteristics observed included spherical to irregularly elliptical morphology of EGTE constituents and high degree of porosity which are supposed to be an important determinant for accelerated wound healing. As these two characteristics are supposed to enhance oxygenation, supply of nutrients, cellular migration and cellular proliferation in wound area (Purohit, ShivDutt et al., 2019; Chuacharoen, Thanida et al., 2019). Reactive Oxygen Species (ROS) play an important role in delayed wound healing, in present In- Vitro study we found that EGTE caused significant amelioration of ROS which is supposed to be an important prerequisite for accelerated wound healing (Syed Muntazir Andrabi et al., 2020, Akbik, Dania et al., 2014). Furthermore, our formulation exhibited significant anti-oxidant and anti-inflammatory activity as can be seen from haemocompatibilty of EGTE at different concentrations with their capability to cause protection against hemolysis. Furthermore, In-Vitro, hemocompatibility assay has been considered as gold standard test for assessing adverse side effects. As per (ASTM, 2000) If any material exhibits more than 5 % of hemolysis it is considered of having adverse side effects and any material exhibiting less than 5 % of hemolysis is considered as biocompatible (Lin, Xinyu et al., 2019).

The compounds present in highest concentrations were studied for their wound healing potential and amelioration of inflammatory and oxidative stress parameters. General characteristics of wound healing components include their potential to cause inhibition of nuclear factor kappa B (NF-κB) pathway (Sophia, Ande et al., 2022). Henceforth in present study we analyzed most prominent components for their ability to cause inhibition of NF-κB. From *In Silico* studies it has been found that compounds having general formula represent by general formula as indicated in *structural formula 1 and 2* (Sophia, Ande et al., 2022). Where X represents connecting group, E aryl group, O oxygen, A hydrogen atom/acetyl group, Rz represents alkyl group and Z represents benzyl group. The components found in highest concentrations in EGTE were found to have almost similar structural configuration as of *structural formula 1 and 2.* In EGTE when we compared structural characteristics of components presented in Supplementary Table 1, we found that almost 13 components exhibited some structural characteristics of *structural formula 1 and 2.*

Diabetes mellitus is characterized by hyperglycemia with other associated dysfunctions, among them delayed and impaired wound healing is prime concern for clinician. Hyperglycemia in DM results in endothelial damage, micro-capillary occlusion, and decreased leukocyte dysfunction which henceforth results in increased risk of infection and delayed wound healing [3]. In present study we used excision wound model in diabetic rabbits for evaluation of wound healing potential of EGTE by topical application, we observed increased wound contraction in EGTE treated rabbits in dose dependent manner compared to control groups. This indicates the presence of significantly more protein content which hastens the wound healing process, which can be appreciated from increased levels of connective tissue markers in granulation tissue extracted from wounds treated with EGTE. Furthermore in current study, EGTE treatment groups exhibited pronounced wound contraction on 5th day post application of ointments compared to vehicle control and distilled water. Hence it can be postulated that EGTE promotes wound healing via induction of proliferation of myofibroblasts, which promotes deposition of extracellular protein network which promotes wound healing in diabetic animal model. These findings are of particular interest for clinician for fabrication of medicinal preparations for treatment of acute wounds in diabetic patients. from results of present study One of the main complications in diabetic wound is addressed which is the persistence/progression of acute wound into chronic phase; hence researchers are in search of drugs which can retard progression of wound into chronic stage (Attoub, Hassan et al., 2011) and current study provide an option for that. The main reason put forward by studies about chronic non healing diabetic wound is immune dysregulation caused by non-resolution of inflammatory phase of wound healing (Li, Wang et al., 2022). From the correlation studies and other biochemical parameters analyzed in current study it may be proposed that EGTE cause resolution of inflammation in diabetic wound which ameliorate immune dysregulation.

The article "Modulation of immune cum inflammatory pathway by earthworm granulation tissue extract in wound healing of diabetic rabbit model" was retracted in 2025. Reasons: unreliable results or conclusions; concerns about the authorship.

In current study, biochemical analysis of granulation tissue revealed significantly elevated levels of hexuronic acid, hydroxyproline and hexosamine in EGTE group compared to levels in vehicle control and distilled water group. Measurement of hydroxyproline and hexosamine has been used as index of collagen turnover and collagen is a predominant protein of the extracellular matrix [48]. In addition to this increased amount of hexosamine content in rabbits treated with EGTE is an indication of collagen fiber stabilization mediated by means of electrostatic and ionic interactions [49]. Henceforth elevated levels of connective tissue markers is an indication of increased cell proliferation and increased synthesis of collagen in rabbits treated with EGTE. The healing potential of incision wound model has been evaluated on basis of granuloma tissue generation, increased granulation tissue occurs because of elevation in levels of collagen which leads to stabilization of wound matrix owing to stabilization of intra and intermolecular cross linking [50]. It can be postulated that EGTE topical application caused modulation in immune cum inflammatory which accelerated deposition of connective tissue parameters, the possible explanation for these finding might be explained on basis of correlation between wound healing percentage observed and inflammatory markers/connective tissue markers.

The results of EGTE having free radical scavenging activity were indicated by significant reduction in free radical and significant increase in levels of antioxidants enzymes. Conversely, free radical mediated cellular damage marker (LPO) were significantly reduced in EGTE groups, apparently significant reduction of LPO levels is an important indication of free radical scavenging activity of EGTE, which ameliorates oxidative damage and henceforth modulates inflammation which plays an important role in wound healing. There are some earlier studies that have reported free radical scavenging activity of crude earthworm tissue extracts, earthworm coelomic fluid extracts and other preparations derived from earthworms, hence based on results of present study it can be postulated that EGTE provides protection to cells and cellular macromolecules under oxidative stress conditions [51]. Researchers have found that free radicals in tissue micro-environment are involved in delayed wound healing in diabetic patients, hence amelioration of oxidative stress by EGTE protect cells from pathological changes initiated by free radicals [52].

The significant elevation in DNA content of granulation tissue in groups treated with EGTE was observed in present study, this indicates presence of active DNA replication and hence active involvement of protein synthesis which is an important prerequisite for wound healing process [53]. Earlier studies have reported that immune and inflammatory cells are actively involved in wound process and TGF β1 has been postulated to play an important role in recruitment of these cells [54]. In-vitro studies have found that TGF β1 inhibits recruitment of inflammatory cells to wound site and promotes synthesis of connective tissue precursors (12) which can be well appreciated from present study, where we observed strongly positive correlation between growth promoters (TGF β1, EDGF and VGEF) and connective tissue markers (hydroxyproline, hexuronic acid and hexosamine). In addition to enhanced production of granulation tissue in EGTE groups, present study we found that EGTE treatment promoted well organized granulation formation (Fig. 8). In addition to this, TGB-β causes differentiation of epithelial cells and hence enhances epithelization in wounded area. Interestingly, accelerated wound closure in EGTE treatment may be attributed to increased expression of TGF-β which causes phenotype switching of fibroblast to myo-fibroblast which helps in deposition of connective tissue matrix in wounded areas [55]. EDGF initiates neo-vascularisation and enhance migration of endothelial cells in granulation tissue; hence organized granulation tissue formation in EGTE treatment may be attributed to neo-vascularisation caused by increased expression of EDGF (Pan, Qi et al., 2022).

The article "Modulation of immune cum inflammatory pathway by earthworm granulation tissue extract in wound healing of diabetic rabbit model" was retracted in 2025. Reasons: unreliable results or conclusions; concerns about the authorship.

However, the levels of IL-6 were reduced in EGTE wound areas and no significant change was observed in levels of IL-6 in control groups. IL-6 is a class of cytokines which possess both anti-inflammatory and pro-inflammatory properties which induces expression of acute phase proteins, henceforth induces inflammation [56]. So it can be postulated that increased levels of IL-6 in wounded area results in delayed healing and hence medicinal preparation which have potential to cause reduction in IL-6 will be effective in accelerating wound healing process. These postulates can be further supported from correlation studies (Fig. 4), where negative correlation was observed between IL-6 with connective tissue markers and growth promoting *m*-RNA markers. Furthermore, EGTE treatment markedly influenced the recruitment of inflammatory cells and hence initiation of inflammation in wounded area as it is demonstrated from diminished levels of pro-inflammatory cytokines like TNF-α, IL-6 and IL-1α in groups treated with EGTE. (TNF) α being an early marker of inflammation produced mainly after an insult in tissue micro-environment ([56]). One of the major takeovers from present study includes an opportunity to evaluate relationship between oxidative stress/growth factors and cytokine levels involved in wound healing process. An interesting finding in present study was an inverse relationship between TNF-α, IL-1β, LPO and IL-6 and growth markers, suggesting possible interaction of these molecules within diabetic wound. These interactions might be involved in pathogenesis hotspots whereby TNF-α, IL-1β, LPO and IL-6 might be having inhibitory effect on the healing process. Earlier studies have well appreciated that TNF-α and IL-1β mediate expression of proteases within wounds, and it is well established fact that micro-environment of diabetic wound is potentially more proteolytic and degradative [57], therefore it might be proposed that TNF-α, IL-1β, LPO and IL-6 might be involved in degradation of enzymatic proteins involved in synthesis of growth markers. Furthermore, formation of biofilms on surface of diabetic wound interacts with host immune system which results in release of pro-inflammatory markers which initiates a vicious circle of further bacterial growth and persistent inflammation in wound micro-environment (Omar et al., 2017). Furthermore, it can be proposed that EGTE treatment accelerates wound healing by modulation of pro-inflammatory response. This proposed mechanistic pathway is of course a speculation, and there is an urgent need of more work to be conducted in-order to decipher this pathway. As pro-inflammatory mediators were significantly decreased in dose dependent manner in EGTE groups, so it can be proposed that EGTE has a potent immune-modulation activity.

The article "Modulation of immune cum inflammatory pathway by earthworm granulation tissue extract in wound healing of diabetic rabbit model" was retracted in 2025. Reasons: unreliable results or conclusions; concerns about the authorship.

## 5 Conclusion

From these findings it can be postulated that EGTE promotes wound healing by scavenging free radicals, dampening of inflammatory pathways, promotion in synthesis of connective tissue framework proteins and enhanced expression of growth promoters. These activities of EGTE may be attributed to the presence of various components present in EGTE. Present study supports the therapeutic utility of EGTE in management of diabetic wound, although further studies are warranted to clearly establish actual role of these types of topical preparations. Although current study postulates probable association between the wound healing and immunomodulatory cum anti-inflammatory properties of EGTE, further studies are required in order to obtain further knowledge for these underlying properties. Based on the characterization studies of EGTE, it may be postulated that there is need of further research to isolate pharmacologically active ingredients from EGTE and evaluate them separately in laboratory animal model.

## Data availability statement

Data will be made available on request.

## Ethical approval

Experiments were performed in accordance with the recommendations of the Committee for Control and Supervision of Experiments on Animals (CPCSEA), Govt. of India. Ethical clearance for the experimental protocol was obtained from the Institutional Animal Ethical Committee (IAEC), Faculty of Veterinary Science & AH, (SKUAST-K), India (No: FVSC/VCC-9/19/439-40).

## CRediT authorship contribution statement

**Ahmed M. E. Elkhalifa:** Writing – review & editing, Funding acquisition. **Sofi Imtiyaz Ali:** Writing – original draft, Conceptualization. **Showkat Ul Nabi:** Writing – original draft, Supervision, Conceptualization. **Imran Bashir:** Writing – review & editing. **Syed Taifa:** Writing – review & editing. **Rabia Rakhshan:** Writing – review & editing. **Iqra Hussain Shah:** Writing – review & editing. **Muzafar Ahmad Mir:** Writing – review & editing. **Masood Malik:** Writing – review & editing. **Zahid Ramzan:** Writing – review & editing. **Mehak Nazar:** Writing – review & editing. **Nusrat Bashir:** Writing – review & editing. **Shubeena Ahad:** Writing – review & editing. **Ibraq Khursheed:** Writing – review & editing. **Elham Elamin:** Supervision, Resources. **Elsharif A. Bazie:** Formal analysis. **Nasser A.N. Alzerwi:** Methodology. **Musaed Rayzah:** Project administration. **Bandar Idrees:** Validation. **Fares Rayzah:** Validation. **Yaser Baksh:** Methodology. **Afnan Alsultan:** Visualization, Validation. **Ahmed M. Alzahrani:** Visualization, Resources.

The article "Modulation of immune cum inflammatory pathway by earthworm granulation tissue extract in wound healing of diabetic rabbit model" was retracted in 2025. Reasons: unreliable results or conclusions; concerns about the authorship.

## Declaration of competing interest

The authors declare that they have no known competing financial interests or personal relationships that could have appeared to influence the work reported in this paper.
